# Impact of the Hormonal Status in Women on Intraoperative Hypothermia during Laparoscopic Gynecologic Surgery when Considering the Fresh Gas Flow Rate: A Retrospective Study

**DOI:** 10.1155/2022/5305165

**Published:** 2022-02-08

**Authors:** Cheol Lee, Juhwan Lee, Gongheui Lee, SeongNam Park, Myeongjong Lee, Hyungtae Kim

**Affiliations:** ^1^Department of Anesthesiology and Pain Medicine, Wonkwang University School of Medicine, 895 Muwang-ro, Iksan 54538, Republic of Korea; ^2^Department of Obstetrics and Gynecology, Wonkwang University School of Medicine, 895 Muwang-ro, Iksan 54538, Republic of Korea; ^3^Department of Anesthesiology and Pain Medicine, Konkuk University Medical School, 82 Gugwondae-ro, Chungju 27376, Republic of Korea; ^4^Department of Anesthesiology and Pain Medicine, Asan Medical Center, University of Ulsan College of Medicine, Seoul 05505, Republic of Korea

## Abstract

Previous studies reported the impact of intrinsic and extrinsic factors on intraoperative hypothermia. However, no clinical study to date has considered the effects of both the phase of the menstrual cycle (an intrinsic factor) and the fresh gas flow rate (FGF) during anesthesia (an extrinsic factor) on the core body temperature and intraoperative hypothermia. This study is aimed at investigatig the effect of the menstrual cycle phase on intraoperative hypothermia when considering the FGF in patients who underwent laparoscopic gynecologic surgery. This study included 667 women aged 19-65 years with menstruation cycles and menopause. The patients were divided into the follicular, luteal, and menopause groups. The primary outcome was the correlations of hormonal status with intraoperative hypothermia. Secondary outcomes included the incidence of intraoperative hypothermia, time to onset of hypothermia, incidence of shivering after anesthesia, and frequency of antishivering drug use in the three groups and risk factors for hypothermia. Overall, the hypothermia incidence was the lowest and the time to onset of hypothermia was the longest in the luteal phase group. At a high FGF, the incidence of hypothermia in the luteal phase group was lower than that in the other two groups (*P* < 0.05). At a low FGF, the time to onset of hypothermia in the luteal phase group was longer than that in the other two groups (*P* < 0.05). The female hormonal status had weak positive correlations with hypothermia at low and high FGF rates. A high FGF in univariate and multivariate analyses, follicular phase and menopause in multivariate analysis, and estradiol and progesterone levels in univariate analysis were risk factors for hypothermia. When considering the FGF, the luteal phase is associated with better outcomes concerning intraoperative hypothermia.

## 1. Introduction

Intraoperative hypothermia is defined as a core body temperature of less than 36°C in patients undergoing anesthesia and surgery [1–6]. An incidence of the condition has been reported between 20% and 90%, depending on the surgical and the demographic factors of the patient [2, 3]. The adverse effects and complications of intraoperative hypothermia include cardiac arrhythmia, wound infection, postoperative pain, shivering, metabolic disturbances, and prolonged hospitalization [1–6].

Normal body temperature varies from person to person according to physiological factors, activities, and external factors [7]. Important risk factors for intraoperative hypothermia include age, sex, smoking, ASA scores, operating room temperature, BMI, preoperative body temperature, type of anesthesia, duration of anesthesia and operation, FGF, and hemodynamic status [2, 6]. To date, there is no strong evidence to identify a single independent variable as a factor that increases the risk of intraoperative hypothermia.

Numerous studies have reported that women's hormonal status affects body temperature control in healthy individuals or patients undergoing surgery under general anesthesia [8–13]. The core body temperature was unchanged from exposure to cold during the follicular and luteal phases. However, the core body temperature in the luteal phase was consistently higher than the follicular phase during general anesthesia and significantly decreased in both the follicular and luteal phases after anesthesia [9, 13].

The mechanism by which women's hormonal status affects the regulated body temperature during the menstrual cycle has been established in humans [8–11]. Progesterone increases body temperature by inhibiting the activity of heat-sensitive neurons, thereby suppressing the mechanism of heat loss. On the other hand, estrogen suppresses the activity of cold-sensitive neurons and stimulates warm-sensitive neurons to suppress the heat preservation mechanism and activates the heat loss mechanism to lower body temperature [8, 10, 11]. Therefore, the phase of the menstrual cycle may affect the core temperature by influencing thermoregulation during general anesthesia [9, 13].

Abundant evidence shows that a low fresh gas flow (FGF) during general anesthesia provides better protection than does a high FGF rate in terms of maintaining the heat and humidity of the respiratory system and minimizing the effects of body heat loss. Thus, the body temperature is higher during low-flow anesthesia than during high-flow anesthesia [14–17].

Previous studies [9, 17] reported the impact of intrinsic and extrinsic factors on hypothermia. However, there was no clinical study that has considered the effects of both the phase of the menstrual cycle (an intrinsic factor) and the FGF during anesthesia (an extrinsic factor) on the core body temperature and intraoperative hypothermia.

We tested the hypothesis that the menstrual cycle phase may affect intraoperative hypothermia differently depending on the FGF (low vs. high) during anesthesia. The present study is aimed at investigating the impact of the menstrual cycle phase on intraoperative hypothermia while considering the FGF rate in patients undergoing laparoscopic gynecologic surgery.

## 2. Materials and Methods

### 2.1. Study Design

This retrospective cohort study analyzed the medical records of all female patients who underwent laparoscopic gynecological surgery under general anesthesia at our hospital from January 1, 2015, to May 30, 2021. Ethical approval for this study (registration number 2021-07-034) was obtained from the relevant institutional review committee.

### 2.2. Patient Selection

For women 19-65 years of age with menstrual cycles or menopause have undergone elective laparoscopic gynecological surgery. It was considered eligible for inclusion in this study. Patients taking medications that could affect cardiovascular function, heat balance, and female reproductive hormone levels or had an implanted device, as well as patients with a history of thyroid disease, autonomic disorders, Raynaud's syndrome, diabetes, or high blood pressure were excluded. Patients with an anesthetic duration of less than 1 hour or converted to open surgery were also excluded. The patients were allocated into three groups: follicular phase (*n* = 232), luteal phase (*n* = 234), and menopause (*n* = 201) groups. The FGF rate during anesthesia was divided into the low flow (≤1 L/min) and high flow (3 or 4 L/min).

### 2.3. Perioperative Management

General anesthesia procedures for all laparoscopic gynecological surgeries performed at our hospital were routinely performed by injecting 1% propofol 2 mg/kg and 1% rocuronium 0.6 mg/kg to induce general anesthesia. Mechanical ventilation of a Primus anesthesia workstation was initiated with a tidal volume of 8 mL/kg and a frequency of 12 breaths/min. The respiratory rate was adjusted to maintain end-tidal CO_2_ at 30-35 mmHg.

The anesthesia was maintained with desflurane concentration, which was titrated to maintain a bispectral index value of 40-60 by adjusting the vaporizer setting to ±1.0 vol%. Before induction of general anesthesia, the patient's core body temperature was measured using an infrared tympanogram. A nasopharyngeal temperature probe was inserted through the nostril, and the probe depth was set to 9.5–10.0 cm for optimal positioning after induction of general anesthesia. Nasopharyngeal temperatures were recorded every 10 minutes until the end of surgery. All patients received a forced-air warming blanket set to supply forced air at 43°C before induction of anesthesia and until surgery was completed.

Upon arrival at the postanesthesia care unit (PACU), the body temperature of all patients was recorded using an infrared tympanic membrane (TM) thermometer. Active warming was applied until discharge from PACU for patients with a TM temperature below 36°C. Postanesthesia shivering was defined as visible and involuntary muscle activity of the face, jaw, head, trunk, and/or extremities. 25 mg of meperidine was administered intravenously to a patient who experienced shivering for more than 10 minutes.

### 2.4. Outcome Variables

The primary outcome was the correlations of hormonal status with intraoperative hypothermia. Secondary outcomes included the incidence of intraoperative hypothermia, time to onset of hypothermia, incidence of shivering after anesthesia, and frequency of antishivering drug (meperidine) use in the three groups and risk factors for intraoperative hypothermia.

### 2.5. Statistical Analysis

SPSS (version 25.0; SPSS Inc., Chicago, IL, USA) was used for all statistical analyses. The groups were compared using one-way analysis of variance (ANOVA) with Bonferroni correction for multiple comparisons or the Kruskal-Wallis test for continuous variables. Categorical variables were analyzed using the Mantel-Haenszel test. The association between variables was analyzed using Phi (*φ*) or point-biserial correlation. We performed univariate and multivariate logistic regression analyses to identify the risk factors associated with inadvertent hypothermia. It was checked whether the predictor variable satisfies the linearity assumption of logistic regression analysis, and variables that did not satisfy the assumption were classified. For model selection, a stepwise forward selection procedure was used to identify candidate predictors with univariate associations of *P* < 0.05. We then evaluated the model for the collinearity problem and investigated key variables for effect correction using interaction terms. Data are presented as mean ± standard deviation, median, or the number of patients (%). We calculated the odds ratio (OR) of the 95% confidence interval (CI). Statistical significance was set at *P* < 0.05 for all analyses.

## 3. Results

From January 1, 2015, to May 31, 2021, a total of 1,200 patients underwent laparoscopic gynecological surgery at our hospital. Of these, 533 were excluded due to incomplete medical records or meeting the exclusion criteria. A final 667 patients were included in the study. (Figure 1).

No significant differences were found between the three groups in terms of FGF, type of surgery, duration of anesthesia and surgery, and amount of infusion fluid. Age and body mass index (BMI) was higher in the menopause group than in the follicular and luteal groups (*P* ≤ 0.01). The TM temperature was significantly higher (*P* ≤ 0.01), but the incidence of shivering after anesthesia (*P* ≤ 0.01) and the frequency of meperidine use (*P* ≤ 0.01) were significantly lower in the luteal phase group than in the follicular group and menopause group (*P* ≤ 0.01). Core body temperature before anesthesia induction and nasopharyngeal body temperature during anesthesia reversal were significantly higher in the luteal group than in the other two groups (*P* ≤ 0.01). The incidence of hypothermia during surgery was lower, and the time to onset of hypothermia was longer in the luteal phase group than in the other two groups (*P* ≤ 0.01) (Table 1).

The luteal phase group had a significantly longer time to onset of hypothermia than the follicular group (*P* ≤ 0.01) and the menopause group (*P* ≤ 0.01) at low FGF. There were no significant differences between the three groups in the incidence of hypothermia during surgery, the TM temperature in the PACU, the incidence of shivering after anesthesia, and the frequency of meperidine use. In contrast, at high FGF, the luteal group had significantly lower intraoperative hypothermia, shivering after anesthesia, and meperidine use and had a higher TM temperature in the PACU than the follicular group (*P* ≤ 0.01) and the menopause group (*P* ≤ 0.01) (Table 2).

At a low FGF, the correlations of estradiol (*r* = −0.19, *P* ≤ 0.01) and progesterone (*r* = −0.25, *P* ≤ 0.01) levels with intraoperative hypothermia were significant and weakly negative. At a high FGF rate, the correlations of the menstrual cycle phase and menopause (Phi [*φ*] = 0.22, *P* ≤ 0.01) with intraoperative hypothermia were significant and weakly positive. Meanwhile, the correlations of estradiol (*r* = −0.27, *P* ≤ 0.01) and progesterone levels with intraoperative hypothermia (*r* = −0.32, *P* ≤ 0.01) were significant and weakly negative (Table 3).

In logistic regression analyses of risk factors associated with inadvertent hypothermia, the OR of the duration of anesthesia was 1.05 (*P* ≤ 0.01) in univariate analysis and 1.08 (*P* ≤ 0.01) in multivariate analysis. The OR of BMI was 0.29 (*P* ≤ 0.01) in univariate analysis and 0.22 (*P* ≤ 0.01) in multivariate analysis. The OR of the FGF rate was 2.85 (*P* ≤ 0.01) in univariate analysis and 53.60 (*P* ≤ 0.01) in multivariate analysis. The OR of the luteal phase was 23.36 (*P* = 0.04) in multivariate analysis. In univariate analysis, the OR of the estradiol level was 0.99 (*P* ≤ 0.01) and that of the progesterone level was 0.89 (*P* ≤ 0.01) (Table 4).

## 4. Discussion

The main finding of this study is that the phases of the menstrual cycle are likely to affect inadvertent hypothermia differently depending on the FGF (low versus high). At high FGF, the incidence of intraoperative hypothermia in the luteal phase group was lower than in the other two groups. At low FGF, the luteal phase group had a longer time to onset of hypothermia than the other two groups.

In the present study, each phase of the menstrual cycle had different effects on the incidence of intraoperative hypothermia, TM temperature, the incidence of shivering after anesthesia, and frequency of antishivering drug (meperidine) use, depending on the FGF. In univariate and multivariate logistic regression analyses of risk factors associated with intraoperative hypothermia, the OR of the FGF rate was greater than that of the menstrual cycle phase. These results imply that the FGF, which is an extrinsic factor, maybe a stronger predictor of intraoperative hypothermia than the menstrual cycle phase, which is an intrinsic factor.

Previous studies have reported a decrease in body temperature with increasing age in women [12]. Core body temperature before induction of anesthesia was higher in follicular and luteal group patients than in menopause patients in this study. However, there was no significant difference in the incidence of intraoperative hypothermia between the follicular group and the menopause group. This may be due to a higher BMI in the menopause group, but there is a conflicting evidence for the relationship of body temperature with BMI [18].

In the present study, risk factors for intraoperative hypothermia were analyzed using univariate and multivariate logistic regression tests. Univariate analysis is the most basic form of the statistical data analysis technique. Univariate analysis techniques are used when your data contains only one variable and does not address cause or effect relationships. Multivariate analysis is a more complex form of statistical analysis technique used when there is more than one variable in a data set [19].

In univariate and multivariate logistic regression analysis, anesthesia time, BMI, FGF, and body temperature before induction of anesthesia were risk factors related to hypothermia during surgery. In a univariate analysis, the effects of estradiol and progesterone levels on intraoperative hypothermia were negligible. Also, in the present study, the correlation between female reproductive hormones, menstrual cycle, and hypothermia during surgery was significant but weak. Therefore, estradiol or progesterone levels may not be strong predictors of intraoperative hypothermia.

The present study is different from a previous study [9] in terms of considering the FGF (low vs. high). The previous study reported the effects of women's hormonal status on core body temperature only at a low FGF during anesthesia. The present study showed that the effect of the menstrual cycle phase on thermoregulation may differ according to the FGF.

This study had several limitations. First, the present study may have selection bias and information bias [20]. In addition, this study has limitations in the generalization of the results due to the small sample size. Studies with larger sample sizes may be needed to clarify controversial results. Second, it could not be confirmed whether the nasopharyngeal upper or middle mucosa was the optimal probe location. Nonoptimally positioned nasopharyngeal temperature probes to achieve significantly different core temperature values from those obtained with optimally positioned probes [21]. Finally, it could not be determined whether all patients in the PACU whose core body temperature was recorded using an infrared TM thermometer had not undergone otoscopy to rule out ear fragments. The auditory readings in the present study may have been influenced by ear fragments and external auditory canal temperature measurements [22].

In conclusion, when considering the FGF, the luteal phase group showed better outcomes than the other two groups in terms of having a lower incidence of hypothermia and a longer time until hypothermia development. However, female hormonal status is not the single independent variable that increases the risk for intraoperative hypothermia. Therefore, extrinsic factors such as FGF should be considered to prevent intraoperative hypothermia in patients who undergoing laparoscopic gynecologic surgery.

## Figures and Tables

**Figure 1:** Consort flow diagram.

**Table 1:** Demographic and perioperative data.

Variables	Groups			
	Follicular (*n* = 232)	Luteal (*n* = 234)	Menopause (*n* = 201)	95% CI
Age (y)	45.9 ± 1.7	45.0 ± 1.5	56.0 ± 3.4^∗^	^∗^vs follicular: 10.5-11.6 ^∗^vs luteal: 10.5-11.6
Body mass index (kg/m^2^)	23.9 ± 2.2	24.1 ± 1.9	24.7 ± 2.2^∗^	^∗^vs follicular: 0.34-1.29 ^∗^vs luteal: 0.07-1.02
Core body temperature before anesthesia induction (°C)	37.0 ± 0.2^†^	37.3 ± 0.2^∗^	36.9 ± 0.1	^∗^vs follicular: 0.25-0.34 ^∗^vs menopause: 0.34-0.43 ^†^vs menopause: 0.01-0.13
Estradiol (pg)	114.2 ± 77.2^†^	136.4 ± 50.2^∗^	6.9 ± 5.1	^∗^vs follicular: 10.35-34.1 ^∗^vs menopause: 117.25-141.86 ^†^vs menopause: 95.02-119.68
Progesterone (ng)	1.2 ± 0.6^†^	11.9 ± 5.3^∗^	0.3 ± 0.1	^∗^vs follicular: 11.44-12.32 ^∗^vs menopause: 10.90-12.32 ^†^vs menopause: 0.15-1.57
Fresh gas flow rate				
Low (≤1 L/min)	112 (48.3)	124 (53.0)	114 (56.7)	
High (3 or 4 L/min)	120 (51.7)	110 (47.0)	84 (43.3)	
Type of surgery				
Laparoscopic subtotal hysterectomy	51 (22.0)	49 (20.9)	45 (22.4)	
Laparoscopic-assisted vaginal hysterectomy	149 (59.9)	142 (60.7)	117 (58.2)	
Total laparoscopic radical hysterectomy	42 (18.1)	43 (18.4)	39 (19.4)	
Duration of anesthesia (min)	96.0 ± 34.9	94.8 ± 35.6	100.1 ± 39.8	
Duration of surgery (min)	66.0 ± 35.0	64.9 ± 36.1	70.0 ± 39.6	
Amount of fluid infused (mL)	950.3 ± 349.9	948.4 ± 3 47.5	1008.7 ± 400.1	
Nasopharyngeal body temperature at anesthesia reversal (°C)	35.9 ± 0.3	36.1 ± 0.3^∗^	35.9 ± 0.3	^∗^vs follicular: 0.078-0.22 ^∗^vs menopause: 0.09-0.24
The incidence of hypothermia	83 (35.8)	50 (21.4)^∗^	69 (34.3)	
Time to onset of hypothermia	70.5 ± 19.5	82.0 ± 25.4^∗^	69.1 ± 22.0	^∗^vs follicular: -15.44-0.05 ^∗^vs menopause: -14.25–1.83
TM temperature (°C) in the PACU	35.8 ± 0.3	35.9 ± 0.3^∗^	35.8 ± 0.3	^∗^vs follicular: 0.08-0.22 ^∗^vs menopause: 0.09-0.06
Shivering after anesthesia	47 (20.3)	26 (11.1)^∗^	44 (21.9)	
Meperidine (25 mg) use	34 (14.7)	18 (7.7)^∗^	29 (14.4)	

Values are expressed as mean ± standard deviation or number (%). ^∗^*P* versus the other two groups. ^**†**^*P* versus the menopause group. PACU: postanesthesia care unit; TM: tympanic membrane; CI: confidence interval.

**Table 2:** Incidence of intraoperative hypothermia and shivering after anesthesia when considering the fresh gas flow rate.

FGF	Follicular (*n* = 232)	Luteal (*n* = 234)	Menopause (*n* = 201)	95% CI
Low				
Intraoperative hypothermia	26 (23.2)	20 (16.1)	24 (21.1)	
Time to onset of hypothermia	83.5 ± 13.5	101.5 ± 15.0^∗^	82.1 ± 17.9	^∗^vs follicular: 6.67-29.41 ^∗^vs menopause: 7.84-31.00
TM temperature (°C) in PACU	35.9 ± 0.3	36.1 ± 0.3	35.9 ± 0.3	
Shivering after anesthesia	18 (16.1)	12 (9.7)	18 (15.8)	
Meperidine (25 mg) use	12 (10.7)	8 (6.5)	7 (6.1)	
High				
Intraoperative hypothermia	57 (47.5)	30 (27.3)^∗^	45 (51.7)	
Time to onset of hypothermia	64.6 ± 19.0	69.0 ± 22.5	62.2 ± 20.7	^∗^vs follicular: 6.67-29.41 ^∗^vs menopause: 7.84-31.00
TM temperature (°C) in PACU	35.7 ± 0.3	35.9 ± 0.3^∗^	35.8 ± 0.4	^∗^vs follicular: 0.06-0.28
Shivering after anesthesia	29 (24.2)	14 (12.7)^∗^	26 (29.9)	^∗^vs menopause: 0.04-0.28
Meperidine (25 mg) use	28 (23.3)	10 (9.1)^∗^	22 (24.1)	

Values are expressed as mean ± standard deviation or number (%). FGF: fresh gas flow rate; PACU: postanesthesia care unit; TM: tympanic membrane. ^∗^*P* < 0.05 versus the other two groups. CI: confidence interval.

**Table 3:** Correlations of menstrual cycle phase and female reproductive hormones with intraoperative hypothermia when considering the fresh gas flow rate.

Fresh gas flow rate	Intraoperative hypothermia	
Low		
Menstrual cycle phase and menopause	Phi (*φ*) = 0.075	*P* = 0.38
Estradiol	*r* = −0.19	*P* ≤ 0.01
Progesterone	*r* = −0.25	*P* ≤ 0.01
High		
Menstrual cycle phase and menopause	Phi (*φ*) = 0.22	*P* ≤ 0.01
Estradiol	*r* = −0.27	*P* ≤ 0.01
Progesterone	*r* = −0.32	*P* ≤ 0.01

**Table 4:** Univariate and multivariate logistic analyses of risk factors associated with intraoperative hypothermia.

Variables	Univariate analysis		Multivariate analysis	
	OR (95% CI)	*P* value	OR (95% CI)	*P* value
Duration of anesthesia	1.05 (1.04–1.06)	≤ 0.01	1.08 (1.06–1.10)	≤ 0.01
Body mass index	0.29 (0.24–0.35)	≤ 0.01	0.22 (0.14–0.33)	≤ 0.01
Fresh gas flow rate	2.85 (2.02–4.03)	≤ 0.01	53.60 (12.64–227.29)	≤ 0.01
Core body temperature before anesthesia induction	0.003 (0.001–0.010)	≤ 0.01	0.00 (0.00–0.002)	≤ 0.01
Menstrual cycle phase	0.95 (077–1.17)	0.63		
Follicular phase (0)				
Luteal phase (1)			23.36 (1.08–504.85)	0.04
Menopause (2)			0.93 (0.22–3.94)	0.93
Estradiol	0.99 (0.992–0.997)	≤ 0.01	1.00 (0.99–1.01)	0.76
Progesterone	0.89 (0.85–0.92)	≤ 0.01	0.80 (0.61–1.06)	0.12

OR: odds ratio; CI: confidence interval.

## Data Availability

The data used to support the findings of this study are available from the corresponding author upon request.
